# Saddle Aortic Embolism Following Recovery From Severe COVID-19 Pneumonia

This article has been retracted.

**DOI:** 10.7759/cureus.18074

**Published:** 2021-09-18

**Authors:** Saeed S Alqahtani, Saleh M Altowygry, Talal E Alebiwani, Mujtaba E Alsaleh, Atheer A Almajed, Mohammed A Alkhamis, Ahmed A Al Abdullah, Mohammed H Almajed, Mohammed E Alhamaqi, Faisal G Aljuhani, Ali A Alsharit, Malak A Alshammari

**Affiliations:** 1 Vascular Surgery, Prince Sultan Military Medical City, Riyadh, SAU; 2 Medicine, King Saud University, College of Medicine, Riyadh, SAU; 3 Medicine, King Faisal University, College of Medicine, Al-Ahsa, SAU; 4 Medicine, Maastricht University, Maastricht, NLD; 5 Medicine, University of Debrecen, Debrecen, HUN; 6 Internal Medicine, Imam Abdulrahman Bin Faisal University, Dammam, SAU

**Keywords:** case report, saddle aortic embolism, saddle embolus, acute low back pain, coronavirus disease 2019 (covid-19)

## Abstract

Coronavirus disease 2019 (COVID-19) is a multi-organ disease with a wide range of manifestations. Coagulopathy is one of the well-recognized complications of COVID-19. We report the case of a 42-year-old man who presented with progressively worsening low back pain of two days in duration. The pain was burning in character, non-radiating, and was not related to movement. The patient had a recent history of severe COVID-19 pneumonia requiring mechanical ventilation and has stayed in the intensive care unit for eight days. He was discharged three days before the acute onset of his back pain. Examination of the lumbar spine was unremarkable. However, lower limb examination revealed coldness and absent pulses bilaterally. The patient underwent computed tomography angiography which revealed complete occlusion of the lower abdominal aorta at its bifurcation. Emergency endovascular treatment was performed to aspirate the clot. The symptoms resolved following the procedure and the patient was discharged on the third post-intervention day. Saddle aortic embolism is a rare life-threatening condition that may present solely with low back pain. The case demonstrated a possible complication of COVID-19 that occurred after the recovery from the acute phase of the disease.

## Introduction

It became evident that the coronavirus disease 2019 (COVID-19) is a multi-organ disease with a broad spectrum of presentations. Hematologic complications are one of the extra-pulmonary manifestations of COVID-19 that carries significant morbidity and mortality. Dysregulation in the coagulation parameters became a well-recognized complication of COVID-19. The hypercoagulopathy in COVID-19 is thought to be related to endothelial injury with subsequent activation of the coagulation cascade [1]. The thromboembolic complications of COVID-19 are broad and range in severity from asymptomatic to organ dysfunction resulting in death. It is worth noting that up to 30% of patients in the intensive care unit may develop venous thromboembolic disease according to initial reports [2]. Additionally, it should be noted that arterial events such as stroke and limb ischemia can also occur in COVID-19. Recently, it has been suggested that the coagulopathy in COVID-19 may extend beyond the period of hospitalization. Here, we present the case of a middle-aged man who developed a saddle aortic embolism following his recovery from severe COVID-19 pneumonia.

## Case presentation

We present the case of a 42-year-old male patient who presented to the emergency department complaining of low back pain for two days before presentation. He reported that the pain was started suddenly while he was playing golf. He described the pain as burning in character and has gradually increased in its severity. The back pain was localized and was not radiating to the lower limbs. He reported that the pain partially improved with simple oral analgesics like paracetamol. The pain was not related to posture or activity and the patient did not identify any exacerbating factors. He scored the pain as 7 out of 10 in severity and it often awakes him from sleep. There was no history of night sweat, fever, weight loss, urinary or bowel symptoms.

The patient reported that this was the first emergency visit for him with this complaint. He did not have any history of chronic back pain. His past medical history was remarkable for hypertension, dyslipidemia, and diabetes mellitus. However, his diseases were well-controlled. Most of his blood pressure measurements were below 140/90 mmHg. His last hemoglobin A1c level was 6.1%. Notably, the patient did not receive the vaccination for COVID-19 and he had a history of severe COVID-19 pneumonia requiring endotracheal intubation and mechanical ventilation. He stayed in the intensive care unit for eight days and was discharged home three days before the onset of his back pain.

The patient has not undergone any surgical operation in the past. His medication history includes metformin 500 mg twice a day, amlodipine 5 mg once a day, and simvastatin 20 mg once a day. He reported good compliance with his medication. He does not smoke or drink alcohol. His family history is remarkable for cystic fibrosis.

On examination, the patient was in distress due to the pain. His vital signs on presentation were as follows: pulse rate of 110 bpm, blood pressure of 124/82 mmHg, respiratory rate of 16 bpm, the temperature of 36.8℃, and oxygen saturation of 97% on room air. Examination of his back did not reveal any deformities and there was no focal tenderness. The range of motion was normal. The pain was not related to the motion. Importantly, the straight leg raise test was negative bilaterally. Examination of the cardiorespiratory system was unremarkable for any abnormality. However, the lower limb examination showed decreased temperature with absent pulses bilaterally.

A basic laboratory investigation revealed a hemoglobin level of 13.9 g/dL, a white blood cell count of 7200/µL, and a platelet count of 350,000 µL. Other biochemical investigations, including renal and hepatic profiles, were normal. However, the D-dimer was slightly elevated with a level of 550 ng/ml (Table 1).

**Table 1:** Summary of the results of laboratory findings

Laboratory Investigation	Unit	Result	Reference Range
Hemoglobin	g/dL	13.9	13.0–18.0
White Blood Cell	1000/mL	7.2	4.0–11.0
Platelet	1000/mL	350	140–450
Erythrocyte Sedimentation Rate	mm/hr.	14	0–20
C-Reactive Protein	mg/dL	5	0.3–10.0
Total Bilirubin	mg/dL	0.9	0.2–1.2
Albumin	g/dL	4.0	3.4–5.0
Alkaline Phosphatase	U/L	62	46–116
Gamma-glutamyltransferase	U/L	40	15–85
Alanine Transferase	U/L	52	14–63
Aspartate Transferase	U/L	40	15–37
Lactate Dehydrogenase	U/L	180	140–280
Blood Urea Nitrogen	mg/dL	14	7–18
Creatinine	mg/dL	0.9	0.7–1.3
Sodium	mEq/L	138	136–145
Potassium	mEq/L	3.4	3.5–5.1
Chloride	mEq/L	99	98–107
D-dimer	ng/mL	550	220–500

In view of the clinical and laboratory markers, the patient underwent computed tomography angiography of the abdomen and pelvis which unexpectedly demonstrated occlusion of the lower abdominal aorta at its bifurcation with extension to both the common iliac arteries (Figures 1-2). Such findings are consistent with aortic saddle embolism. Subsequently, the 12-lead electrocardiography showed a normal sinus rhythm and the transthoracic echocardiography showed no intracardial thrombus.

**Figure 1:** CT angiography at the level of the aorta Computed tomography angiography image demonstrating a filling defect in the infrarenal aorta (arrow).

**Figure 2:** CT angiography at the level of common iliac arteries Computed tomography angiography image demonstrating complete opacification of the common iliac arteries bilaterally (arrows).

Anticoagulant therapy with low-molecular-weight heparin was initiated immediately following the diagnosis. The patient was prepared for emergency endovascular treatment. A bilateral femoral artery catheterization was performed. The thrombus was completely aspirated by the guiding catheter. The patient tolerated the procedure without any complications. His symptoms showed significant improvement after the procedure. He was discharged on the third post-intervention day and was kept on aspirin as prophylaxis.

## Discussion

We presented the case of a middle-aged man with recent recovery from severe COVID-19 who presented with a progressively worsening lower back pain due to an acute saddle aortic embolism, which is a very rare clinical condition. Saddle aortic embolism is a potentially life-threatening condition with a reported mortality rate between 25% and 75% [3]. The causes of death include multiorgan failure and severe reperfusion injury with electrolytes disturbances. Early recognition and management of this condition define the prognosis [4].

Almost in three-fourths of cases, the source of aortic saddle embolism is cardiac in origin. Atrial fibrillation and myocardial infarction are the most frequent cardiac causes [4]. In our patient, the electrocardiography findings revealed normal findings. However, this does not exclude the possibility of a transient previous arrhythmia precipitating the thromboembolic event.

In a retrospective study by Ding et al. [3] involving 18 patients with aortic saddle embolism, all patients were found to have acute bilateral lower limb pain. The clinical presentation in our case was very atypical as the patient presented solely with acute lower back pain. However, the coldness of the lower extremities and absent distal pulses were suspicious for an ischemic etiology. Further, paraplegia could be the presenting symptom of aortic embolism giving the impression of neurologic disease.

While ultrasound examination aids in making the diagnosis, CT angiography remains the modality of choice. The extent of the thromboembolic disease varies and may include the renal or femoral arteries. The management of aortic saddle embolism includes surgical embolectomy, medical thrombolysis, and endovascular treatment. The present case demonstrated the feasibility of the endovascular approach in such patients [5].

## Conclusions

Saddle aortic embolism is a rare life-threatening condition. Physicians should consider it as a differential diagnosis of acute lower back pain in patients with absent lower extremities pulses. If available, endovascular treatment remains a feasible and successful management approach. The case demonstrated a possible complication of COVID-19 that occurred after the recovery from the acute phase of the disease. Further evidence is needed on the possible use of thromboprophylaxis in patients recovering from severe COVID-19 pneumonia.
